The article "Identification and Analysis of Key Barriers of BIM Application for Small- and Medium-Sized Fire Protection Enterprises" was published in 2022. Journal: J Environ Public Health.

# Identification and Analysis of Key Barriers of BIM Application for Small- and Medium-Sized Fire Protection Enterprises

**DOI:** 10.1155/2022/9240224

**Published:** 2022-09-29

**Authors:** Hui Liu, Ruixiang Zhang, Hang Zhang, Hongbing Jiang, Qianqian Ju

**Affiliations:** Department of Engineering Management, School of Management, Zhengzhou University, No. 100 Science Avenue, New High-Tech District, Zhengzhou, Henan Province 450001, China

## Abstract

The application of Building Information Modeling (BIM) in fire protection discipline has been sufficiently proved to be useful, but has encountered many barriers in China. Among which, small- and medium-sized enterprises (SMEs), which are considered sensitive to adoption costs and external funding support, play a critical role in the BIM adoption process in fire protection discipline. Therefore, identifying and analyzing the barriers of BIM application are essential to help small- and medium-sized fire protection enterprises to overcome these barriers. In this study, semantic analysis, which includes word frequency analysis and coword analysis, based on literature review was utilized to identify the main barriers. 20 main barriers, which were classified into software, people, organization, and environment group, were obtained. Then, Interpretive Structural Modelling (ISM) approach and Cross-Impact Matrix Multiplication Applied to Classification (MICMAC) analysis were utilized to hierarchically analyze and categorize the main barriers of BIM application in Chinese SMFEs. The findings revealed that the lack of external support and the lack of BIM laws and regulations applicable to fire protection discipline are the key barriers in general for the application of BIM in SMFEs. For the barriers at the enterprise level, through further analysis and discussion based on barriers in the people and organization clusters, the lack of funding support for proper BIM training and the lack of organization culture support were concluded as the key barriers of BIM application inside the scope of SMFEs. According to 80-20 principle, more effort should be focused on the key barriers to gain maximum management effect. The research result categorizes the barriers for easy intervention of fire protection enterprises' managers and policymakers. It contributes to the nascent studies of BIM application and provides guidance for the application of BIM in fire protection discipline.

## 1. Introduction

In the global construction market, with the development of informatization and industrialization, fire protection has received more and more attention. Over the past few years, many considerable fire accidents happened in construction building sites were reported. Many construction sites do not contain a permanent fire protection system, and even some current fire protection systems only consist of fire extinguishers. Traditional safety planning lacks a justified approach for the firefighting equipment installation planning in the construction site. Low efficiency of fire protection engineering seriously hindered the sustainable development of construction industry. As the largest construction market worldwide [1], China's construction industry is facing the challenges caused by rising labor cost, sustainable development requirements, etc. [2].

The advent of Building Information Modeling (BIM) is claimed to offer a promising opportunity to harness the effectiveness and efficiency of the fire protection engineering. BIM is a digital representation of a constructed facility [3] and offers an important platform of “integration” [4], which is likewise critical for the design of fire protection engineering. Accordingly, Kincelova et al. [5] proposed a BIM-based fire inspection approach for high-rise wood structure building. Bi et al. [6] acclaimed a BIM-assisted construction fire safety planning method. Digital fire control system can be designed and implemented by combining BIM and 3D-GIS technology. Chen et al. [7] constructed a BIM AR FSE (augmented reality fire safety equipment) system, which provides highly comprehensive, mobile, and effective access to fire safety equipment information. Nevertheless, the actual deployment and implementation of BIM in fire protection engineering still confronts with marvelous barriers which hinder the fire protection discipline to utilize the benefits of BIM to realize effectiveness and efficiency improvement. Nowadays, more and more researchers realize the importance of exploring the application barriers of BIM in construction enterprises and projects. Relevant studies indicated that BIM facilitates the design and visualization of buildings, as well as the detection and modification of conflicts in building models, and the integration and collaboration of relevant personnel. However, the popularity of BIM in fire protection enterprises is still not high. In addition, SMEs are the main components of the fire protection discipline. Comparing with large enterprises, they are more sensitive to costs, and their talent capabilities are at a disadvantage. Therefore, it is necessary to study the small- and medium-sized fire protection enterprises alone.

Therefore, this study aims to identify and hierarchically analyze the application barriers of BIM for small- and medium-sized fire protection enterprises (SMFEs) in China. Three subobjectives are to be achieved: (1) to discover the main barriers of BIM application in China's SMFEs, (2) to assess the interrelationships between these barriers and prioritize these barriers based on their interrelationships, and (3) to analyze the key barriers and classify them according to their independence.

By doing so, the contributions made by this study are four-folded: (1) it bridged the gap of systematic research on the barriers of BIM application in SMFEs, (2) it introduced an innovative barrier identification method that formed the main barriers, (3) fire protection enterprises can develop coping strategies to promote BIM application by controlling the key barriers and avoiding derivative incidents based on the recognized interactions of BIM application barriers, and (4) dynamic barriers and categories help strategy-making of policymakers and managers.

## 2. Research Background

### 2.1. BIM for Small- and Medium-Sized Fire Protection Enterprises

Fire protection discipline is an important part of the construction industry. According to the report released by Autodesk, BIM is mostly associated with design and preconstruction, it absolutely benefits every phase of the project life cycle [8]. Fire construction contractors, the ones specialized in the installation of fire protection facilities, water and electricity pipelines, etc. have realized that the application of information technology (IT) is crucial to their success. On the one hand, by utilizing BIM, fire protection discipline is capable of getting involved in the design stage and can estimate the material costs and staff power accurately. Besides, they can evaluate the system load and supply capacity of the fire-fighting equipment supplier before installing in the project. On the other hand, integrating BIM data with resource planning can reduce errors and enhance the overall management of inventory for fire protection enterprises. In addition, combining BIM with building fire safety management system could accelerate the establishment of life cycle cost-effective assembling processes for construction projects.

So many advantages of BIM technology have been discovered in fire protection discipline. However, the current status of BIM application in the field of fire protection is not very good. BIM application in software, knowledge, investment and the legal environment is still facing many dilemmas. Research pertaining to BIM in the fire protection discipline have emerged only recently. Thus, it is necessary to systematically sort out and analyze the barriers for BIM application in fire protection discipline. According to the definition given by the Ministry of Industry and Information Technology of China, small, medium, and micro enterprises are ones with operating income of less than 800 million yuan or total assets of less than 800 million yuan. Among them, medium-sized enterprises with operating income of 60 million yuan and above and total assets of 50 million yuan and above; small enterprises with operating income of 3 million yuan and above and total assets of 3 million yuan and above. Among China's fire protection enterprises, SMEs account for about 28%, occupying a relatively large ratio. Besides, comparing with large enterprises, the composition of small- and medium-sized enterprises is more complex. They will encounter more barriers such as costs and lack of external funds; on the other hand, the functions of small- and medium-sized enterprises in BIM cannot be ignored. Large enterprises can participate in the formulation of BIM standards, while small- and medium-sized enterprises are the key subjects in the application of BIM standards, which is a more critical issue for the widespread application of BIM in fire protection discipline. Therefore, identifying and analyzing the barriers of BIM application in Chinese SMFEs are extremely critical to promote the process of BIM application in fire protection discipline.

### 2.2. Barriers of BIM Application

Application barriers of BIM have always been a hot topic. Researchers from different disciplines tend to study related barriers for BIM application. BIM can facilitate the delivery of prefabricated construction. Wu et al. (2020) have studied the BIM application barriers of industrialized building construction systematically, which concentrated more on data integration and information models [9]. Tan et al. [10] studied the barriers to BIM implementation in China's prefabricated construction. Durdyev et al. [11] offers a prioritized list of barriers that are inhibiting industry-wide adoption of BIM during the facility management phase. Chiu et al. [12] also offered the barriers on achieving wider adoption of BIM in building services engineering.

Amount of research on the barriers of BIM for SMEs is also raising, Li et al. [13] studied the main challenges hindering the adoption of BIM in SMEs. Abdullahi et al. (2020) evaluated and investigated the dynamics of the barriers of BIM adoption from the perspective of SMEs in developing countries [10]. For specialty contracting SMEs, Poirier et al. (2014) studied the radical innovation process behind the adoption and implementation of BIM, which provides a meaningful perspective for the research on the incentives of BIM application in fire protection discipline.

There are many studies focusing on BIM application barriers in the construction industry, nevertheless, the study with respect to BIM application barriers in fire protection discipline is still scarce. Although Kincelova et al. [5] pointed out some meaningful barriers when SMFEs applied BIM in projects, systematic and comprehensive research on barriers to BIM application in fire protection discipline, especially the SMFEs, is still lacking.

## 3. Methods

In order to fulfill the research objective, a three-step method was utilized in this study, and the detailed research procedure, as shown in Figure 1, will be demonstrated as following.

### 3.1. Data Collection

The goal of the data collection was to find literature regarding barriers that hinder the application of BIM in fire protection discipline. The data collection started with a literature search. Scopus, WoS, and Google Scholar engines were selected as the target databases, “BIM”, “barrier”, “obstacle”, “application”, “application”, and “implementation” were used as keywords for literature search. There are 45 articles found in the above process. The abstracts of each paper were read by the research team members in order to screen out articles relevant to these two topics: BIM application barriers in SMEs and fire protection discipline.

After the search was completed, 20 articles were selected as the basis for the next step of barrier extraction. In the barrier extraction, the lists of barriers or subheadings about the barrier in the selected literature were extracted one by one. After filtering by removing duplicates, each barrier was filled in each row of the first column of the table, resulting in a total of 355 barriers. The results were summarized in Totalbarrier.xlsx.

### 3.2. Identification of the Main Barriers

Semantic analysis is the process of drawing meaning from text. It allows computers to understand and interpret sentences, paragraphs, or whole documents by analyzing their grammatical structure and identifying relationships between individual words in a particular context. In this study, semantic analysis was applied for barrier identification. To be specific, word frequency analysis and associated coword analysis were used to complete the process of transforming barriers texts to keywords abstraction to main barriers list. The detailed procedure is shown in Figure 1.

#### 3.2.1. Word Frequency Analysis

Word frequency analysis is a statistical analysis of the number and percentage of words in a text. It is an important tool for text mining. It determines keywords and their trends by calculating the frequency of words appearing in the text. In this study, word frequency analysis was used to analyze the barriers from the literature. These barriers are usually expressed in the form of a single statement, and similar barriers often have the same keywords. For example, BIM software cost is a high frequency barrier, so the keywords like “software”, “cost”, and “difficult to pay” and other keywords may appear frequently. Therefore, this paper finds out the high frequency keywords of these barriers and then classifies these words simply according to their meanings.

In the process of word frequency analysis, Totalbarrier.xlsx is used to create a plain text file containing only barriers. The specific method is to copy and paste directly from the first column of the table into the text document, and ensure that each barrier occupies a separate line. This operation is more convenient for Nvivo analysis. Then, the high frequency words in the text were extracted using the word frequency function in the Nvivo software. The result is shown in Figure 2. As is shown in Figure 2 that “software” is the word with the highest frequency, and other words with similar frequency are “cost”, “technology”, “change”, “standard” “projects”, etc. These high-frequency words are continually found among the barriers studied in the literature and can often be used as a proxy for the classification of all barriers (these words have higher correlation with other words). After above extraction, the keywords were classified into four main sections according to word frequency result and logical juxtaposition: software, people, organization, and environment. The classification result is shown in Table 1. According to Table 1, the software section, including cost, pay, and data, accounts for 39% of the total barriers, barriers in the organization section account for 74%, barriers in the people section account for 43%, while barriers in the environment section account for 64%. Next, according to the keywords of each section given by the classification results, the search feature of Excel was applied to create a plain text document of the barrier entries related to each section, respectively, and then, the text document was input into the Nvivo to conduct the categorized word cloud and their frequency, which is shown in Figure 3. According to Figure 3, cost, complexity, hardware, data, and expert have a larger weight in software section, which means these words are most dominant among the barriers under software classification. Likewise, knowledge, stakeholders, benefits, reluctant, and collaboration are significant in the people section. Training, time, collaboration, cost, investment, and learn are most important in the organization section, and standards, resources, demand, model, contract, interest, and government are given priority in the environment section.

#### 3.2.2. Associated Coword Analysis

As to the specific description of each section of barriers, the word frequency analysis alone is not sufficient, therefore, the associated coword analysis was used to form the final main barriers list.

The association rule is a knowledge mode that describes the law of the simultaneous occurrence of items in a thing, that is, the emergence of quantified data A affects the emergence of B. The coword association analysis takes this as the principle, and the dependence relationship between the subject words is revealed through the correlation statistical method. For example, for the keyword cost, the related modifiers include high, highly, etc., indicating that the cost is high, not low, or an appropriate cost.

The COOC software was utilized for obtaining keyword cooccurrence matrix. The rows and columns in the matrix represent any two keywords and the number in the cell indicate the cooccurrence frequency of the two words in the barrier total list. The matrix was then modified in Excel to output the node file, which contains the keywords and their frequencies, and the edge file, which includes the keyword cooccurrence relationships (the direction was set to “undirected”). The node file and edge file were imported into Gephi software. The visualization map of the interrelationships between barriers was achieved (shown in Figure 4). However, it is difficult to express the coword relationships among the classified barriers groups. The result shows that there are different ways for keywords linkage to those in Table 1 and the others. The other keywords have the characteristic of forming sentences with the keywords in Table 1, which allows the analysis of the specific formulation of the barriers in each section (e.g., the other keyword like “match” is more likely to be combined with the “hardware” in Table 1. The sentence they formed means *It is hard to match the BIM software and hardware in fire protection discipline*). After importing the classification results in Table 1 into Gephi analysis, the categorized Gephi network was achieved (as shown in Figure 5). Through visual analysis, it can be clearly observed whether the keywords match with one or more related cowords, as shown in Table 2. Their combination forms a complete semantics of barriers, some of them consist of several keywords or one main barrier keyword, and some of them have only one main barrier keyword with another one keyword. For example, “cost” and “high” consist a barrier as “software cost is high”, and “knowledge” and “experience” formed a barrier as “people is lack of knowledge and experience in BIM application”. In addition, some adjectives and common verbs in total list of barriers, such as “lack” and “available”, have been retained as derivatives for combined semantics.

#### 3.2.3. List of the Main Barriers

In addition to above research, we combined interview in the main barriers. For the purpose of getting practical opinions about barriers, we conducted an oral interview. A total of 20 experts suitable for this survey were contacted through telephone or email. The experts were chosen based on their professional background, experience, and ability to ensure that they have extensive knowledge and experience in the field of fire protection discipline. Finally, five experts agreed to participate in the survey, and their profile is shown in Table 3. Most of the time, we conducted interviews by phone with experts located in Shanxi, Anhui, Henan, and Jiangxi. Another expert in Henan was interviewed in person, and the interview time was in the fall of 2021 or later. In the oral interview, we asked some interesting questions, as follows:

1. Do you think our barrier factors are more comprehensive?
2. Do you have any other comments on the barriers to BIM application in fire protection enterprises?

We have received valuable feedback from which we have summarized several barriers that were not on the initial list of barriers but were very important.

In the end, combining the results of semantic analysis and interview, 20 main barriers of BIM application in SMFEs were identified, which is demonstrated in Table 4. Table 4 lists the references of each barrier, as well as the specific explanations of the four sections.

### 3.3. Analysis of the Main Barriers through ISM and ICMAC Approach

ISM method was applied in this study for level partition of the main barriers, and the key barriers were identified through MICMAC matrix. The analyzing procedure is shown in Figure 6.

#### 3.3.1. Establishment of Initial Reachability Matrix

The initial data for ISM method was obtained through interviews with experts of fire protection discipline. The interview questionnaire involved basic information about the experts and the relationships between the barriers. After sorting, the structural self-interaction matrix (SSIM) of the selected barriers was generated. The accessibility judgment and processing of the SSIM was conducted for the reachability matrix. Accordingly, the main barriers were hierarchically analyzed. After that, the MICMAC analysis was applied to classify the barriers into four categories, independence, dependency, linkage, and autonomous, based on the calculation of driving powers and dependence powers represented in the reachability matrix. Among which, the independence barriers were considered as the key barriers in this study.

In the process of data collection, we conducted an interview with selected five experts by phone or in person, as shown in Table 3. Five experts were acceptable to be sufficient in BIM-related ISM analysis; for example, Farooq et al. [23] investigate BIM implementation barriers use ISM approach with five responses. Eight expert interviews have been conducted in the study of Abbasnejad et al. [22]. Onososen et al. (2022) received fourteen responses serving for a wider area of investigation. All five experts were asked questions about the relationship between each two barriers, the results of which were transformed into the SSIM, as shown in Table 5. In this study, the interrelationships between barriers *i* and *j* were represented by four symbols:

1. *W* refers to “barrier *i* can result in barrier *j*”
2. *X* refers to “barrier *j* can lead to barrier *i*”
3. *Y* refers to “barriers *i* and *j* can lead to each other”
4. *Z* refers to “barriers *i* and *j* are not related”

In cases when different experts made different judgments towards the relationship of two barriers, the “minority gives way to the majority” principle was applied in order to determine the interrelationships.

In this way, contextual relationships between the 20 barriers were constructed from feedback. For further calculation and analysis, *W*, *X*, *Y*, and *Z* were then converted into 1 and 0, consequentially, the developed SSIM was converted into a binary matrix. An initial reachability matrix was established, which is shown in Table 6, explaining the pairwise interrelationships among the 20 barriers, according to the rules given in Table 7.

#### 3.3.2. Establishment of Reachability Matrix

Transitivity is one of a basic assumption of ISM method. If factor *i* affects factor *j* and factor *j* affects factor *k*, then factor *i* will definitely affect *k*. The reachability matrix can reveal whether there is a path connecting one factor to another. If the cell (*i*, *j*) in the reachability matrix is equal to 0, then there is no direct or indirect relationship from factor *i* to factor *j*. According to this principle, the reachability matrix can be computed according to the following Boolean rules:

(1) $$\begin{array}{c} R={\left(A+I\right)}^{r}={\left(A+I\right)}^{r-1}\neq {\left(A+I\right)}^{r-2}\neq \;\neq \left(A+I\right),\;r\leq 19. \end{array}$$

In Equation (1), *A* is the initial reachability matrix, *I* is the unit matrix, and *R* is the reachability matrix. According to Equation (1), the reachability matrix is obtained with open-source online platform (https://spssau.com/indexs.html) by input and output, as shown in Table 8. Then, the driving power and dependence power of each barrier were determined according to the number in each row and column, respectively, in reachability matrix.

## 4. Results

### 4.1. Hierarchical Structure and Level Partitioning

Reachability sets and antecedent sets are extracted from the reachability matrix [35]. Reachability sets for a specific barrier in the study include identified barrier variables and several other barrier variables that it may assist in achieving. Antecedent sets comprise the barriers identified and the barriers that they may contribute to achieve. Consequently, the intersection of these sets is obtained for all barriers and noted as intersection sets. The level partition can be seen in Table 9. Then, a conical matrix was made by sorting the reachability matrix by level partition to help the construction of the ISM model. Next, the structural model or digraph (as shown in Figure 7) was made according to level partitioning and the relationships between criteria in the reachability matrix. Following that, the digraph in Figure 7 was transferred into ISM model, as shown in Figure 8, by changing the element node with barrier.

As shown in Table 9 and Figure 8, the 20 main barriers were partitioned into five levels. At the bottom level, namely, level V, located the lack of external support such as funding from local government (B17) and the lack of BIM laws and regulations applicable to fire protection discipline (B15), which were taken as the root barriers or the key barriers for BIM application in SMFEs. Barriers 1~4, 7, 9~11, 14, 16, and 19~20 placed at level IV. Among which, there were similar situations (relationships with other barriers) happen to barriers 1~4, 9~11 and 14, 19~20. Accordingly, in purpose of making the hierarchical model easy for users to analyze, through brainstorming and literature review, we combined the above barriers into five clusters: software and technology-based barriers (consist of B1~B4), internal enterprises BIM barriers (consist of B9~B11, B14), external guidance barrier (consists of B19~B20), and B7 and B16. At the level III were B12 and B18, which involve the BIM-related knowledge and skills of staffs in the enterprise and the requirement of BIM application in guidance and standard of industry and appropriate regulatory rules. The barriers 5, 8, and 13 were placed at level II. It can be interestingly found that B5 (top managers' coordination and scheduling capabilities) and B13 (instability of business development in organizational culture) possess similar relationships with other barriers, e.g., barriers at the level III and level I. It may be because that B5 and B13 are barriers related to the administrative issues related to the BIM application in SMFEs from different perspectives. Lastly, B6 is located at the top level, namely, level I, in the partition diagraph.

### 4.2. MICMAC Analysis

As explained from previous studies [36, 37], MICMAC is built on multiplication properties of matrices. The MICMAC analysis was computed using the dependence power and the driving power for each of the barriers as shown in Table 7. The dependence power and the driving power are the sums of all values in a row and a column, respectively, for a barrier depending on the final reachability matrix table. The dependence power and driving force are used to plot the diagram (Figure 9), which contains four categories as following.

- Independent factors

Barriers in this category have high driving power, but low dependence power, which is used to be the key factors in this study. The barriers in this category are lack of BIM laws and regulations applicable to fire protection discipline and lack of external support such as funding from local government. These barriers should be prioritized, and relevant managers should try to avoid or minimize the negative impact of these barriers.

(ii) Linkage factors

The barriers in this cluster are high in both driving power and dependence power, making it unstable. The barriers in this category are high cost of BIM software, lack of domestic-oriented BIM tools, high cost of supporting hardware upgrades required, lack of suitable simulation models for fire protection engineering, lack of knowledge and experience in applying BIM, lack of funding support for proper BIM training, lack of organizational culture support (a shared vision for the BIM application), ambiguity about the benefits of BIM, lack of investment in BIM experts, lack of demand for BIM application from clients, lack of pilot projects for BIM applied in fire protection projects to learn from, and lack of BIM contract standards suitable for fire protection enterprises. These barriers are considered the second most critical barriers that companies should make their efforts on.

(iii) Dependent factors

Factors in this group have low driving power and high dependence power that makes it vulnerable to change. The criteria in this category are top managers are not adapting to the new requirements for coordination and scheduling capabilities, low level of cross-functional coordination and collaboration, lack of knowledge and experience in cross-organizational collaboration, difficulty accepting the instability of business development brought by changes in organizational structure, and lack of appropriate government regulatory measures. These barriers show indirectness to the core problem. What companies should consider is to focus on the effectiveness of improvement measures on these barriers.

(iv) Autonomous factors

Because of the low driving power and dependence power of the barriers in this group, the barrier in this category can be separated from the assessment system. No barrier factor is located in this category.

In the end, we conducted informal interviews by phone or email. The interviews included thanking the respondents and asking them for their views on the results of the analysis. Although some relationships differed from the content of the initial response for some experts, but generally they are acceptable. Experts gave a reasonable judgment of the results, either verbally or by mail.

## 5. Discussions

From the results of ISM and MICMAC analysis, government, project owners, consultants, designers, contractors, and software vendors are the key participants and real executors in applying BIM technology. They must work collaboratively to improve the effect of BIM application. Extensive effort should be focused more on the root barriers, the roots on the level V and level IV in the partition diagraph, which are also located in the independent and linkage clusters as shown in Figure 9.

Results of the MICMAC analysis revealed that the environmental barriers are the most influencing barriers for BIM application in fire protection discipline. Among which, the most critical barriers were B15 and B17. The lack of BIM laws and regulations applicable to fire protection discipline (B15), especially the limited funding and technology assistance of government to make BIM suitable for fire protection enterprises (small- and medium-sized ones in particular) in China's local context, is the most fundamental barrier in the hierarchy. This finding suggests that the application of BIM in fire protection enterprises should seriously consider the unique external environment for SMFEs. The lack of external support such as funding from local government (B17), which located on the bottom level of the level partition diagraph (as shown in Figure 8), relates to the laws and regulations supporting for fostering a suitable cooperation environment. These barriers were clustered in the independent cluster in the MICMAC analysis and can be perceived as the root barriers that have direct or indirect causal relationships to the other main barriers. Thus, administrative efforts should be prioritized to them so that to use minimum effort while produce maximum effects according to the 80-20 principle. The findings of this study are consistent with the research result of Li et al. [13] that lack of BIM laws and regulations, and shortage in funds and talents for BIM application in SMFEs directly led to the failure of most enterprises to successfully work with it. Poirier et al. [14] highlighted the strong need for clear policy for supporting BIM application at the industry level because this could lead to a chaotic resource system and economic losses, which is significantly for most SMEs.

Barriers on the level IV of Figure 8 were also clustered in the linkage cluster in the MICMAC analysis. Barriers in the linkage cluster are easily influenced by barriers in the independent cluster while changes in these barriers can strongly influence the barriers in the dependent barriers, which located on the levels I, II, and III (as shown in Figure 9), and are clustered in dependent cluster (as shown in Figure 9). Therefore, these barriers require to be managed and controlled carefully to reduce the negative influence on BIM application in SMFEs. Specifically, barriers in this group include external guidance barriers (lack of pilot and standards for BIM application (B19, B20)), internal enterprise BIM barriers (insufficient training, culture, knowledge, and investment within enterprise (B9-B11, B14)), software and technology-based barriers (high cost, lack of domestic-oriented tools, hardware upgrades barrier, and lack of suitable model for projects (B1-B4)), and the lack of knowledge and experience in applying BIM (B7).

Furthermore, in order to provide more practical recommendations based on the findings of this research, barriers inside the scope of the SMEFs were analyzed specifically as following.

Barriers located in the group of “people” and “organization”, which are barriers especially focused inside the scope of SMFEs, were separated for further analysis by ISM. The new level partition inside the scope of SMFEs, as demonstrated in Figure 10, shows that the resistance to the new technology change is mainly due to personal ability limitation and their concerns about the working environment change. Fundamentally speaking, in order to promote the reform of BIM application within SMFEs, more attention should be paid to B7, B9, B10, and B11, which means to promote the BIM application in SMFEs through changing the enterprise culture, increasing the investment in BIM training, and improving the level of BIM knowledge inside the enterprise, among which the key barriers inside the scope of SMFEs of the BIM application are the lack of funding support for proper BIM training (B9) and the lack of organization culture support (B10), which echoed the claim of Vidalakis et al. (2020) and Awwad et al. [38] that the financial support of BIM determines the popularization and training of BIM in the enterprise [39].

## 6. Conclusions

Although there have been extant studies with respect to investigating the application barriers of BIM in the construction industry, the main thrust of this study is that it focuses on the fire protection discipline, where the BIM application is weaker.

To identify and analyze the barriers for BIM application in SMFEs, the research methods adopted in this study were suitable and effective. First, this study innovatively utilized the semantic analysis, which consists of word frequency analysis and coword analysis, based on traditional literature review for the main barriers identification. In this way, the identification process can be more objective and scientific. In the end, 20 main barriers, which were grouped into software, people, organization, and environment groups, were identified for further analysis.

Second, the ISM combined with MICMAC were applied for barriers analysis. On the one hand, the interactions between BIM application barriers are easily acquired through interview, while the single evaluation of the traditional Likert scale is more subjective and difficult to guarantee the authenticity under multifactors. On the other hand, analysis through ISM combining the MICMAC method can partition barriers into different levels and divide them into four separated categories with various management priorities.

In the end, the key barriers were selected (the barriers located on the lower level, level V and level IV, in the partition diagraph (see Figure 8) and barriers located in the independent and linkage clusters (see Figure 9)). It was shown that the external (government or industry pioneers) supports and the lack of BIM laws and regulations applicable to fire protection discipline were perceived as the most critical barriers for BIM application in SMFEs. Key barriers play a leading role among the other main barriers. According to the Pareto principle (merely about 20% of the variables control and 80% of the situation), extensive effort should be focused more on the root barriers, the roots on the level V and level IV in the partition diagraph, which are also located in the independent and linkage clusters as shown in Figure 9.

The study also addresses dynamic BIM application barriers from the internal enterprise perspective, which has rarely been further analyzed in existing research. It revealed the key internal enterprise barriers BIM application in SMFEs are the lack of funding support for proper BIM training (B9) and the lack of organization culture support (B10). The findings underscore that the SMFEs can drive BIM adoption through internal will and actions such as organization-wide reforms. Moreover, on the contrary, the improvement of management's ability is not as urgent as the improvement of employees' knowledge and skills related to BIM application.

The contribution made by this study is firstly bridging the gap of systematic research on the barriers of BIM application in SMFEs. This study promoted an innovative combination of semantic analysis method for barrier identification, which is more scientific and objective. Moreover, the partition of the barriers prioritizes the focus of efforts to apply BIM in the fire protection discipline. According to the result, the mechanisms by which these barriers affect BIM application in SMFEs are elucidated, which enhances the understanding of BIM application and can accelerate the BIM knowledge popularization process in SMFEs and the dynamics of the barriers and categories for easy intervention by policymakers and stakeholders.

Regardless of the contributions of this study, it has also created a need for further exploration. For example, although the experts selected for data input for the ISM and MICMAC analysis in this study were knowledgeable and with sufficient BIM experience, the number of the experts is small. Thus, further study with a bigger sample should be conducted to validate the result of this research. Besides, the data collected was from China, albeit the barriers identification and analysis process has considered the characteristics of the SMFEs on a general level, research aiming at a wider scope is also necessary. The identification and analysis method combination and the barriers framework proposed in this study can serve as a solid departing point for further exploration on BIM application barriers in fire protection discipline.

## Figures and Tables

**Figure 1:** The detailed research procedure of this study.

**Figure 2:** Word cloud and frequency of the barriers.

**Figure 3:** Categorized word cloud and their frequency.

**Figure 4:** Uncategorized Gephi network.

**Figure 5:** Categorized Gephi network.

**Figure 6:** Process of the hierarchical analysis of BIM application barriers of SMFEs based on ISM and MICMAC method.

**Figure 7:** Interrelationships between 20 barriers.

**Figure 8:** Level partition of the main barriers of BIM application in SMFEs.

**Figure 9:** Classification results of MICMAC analysis of the main barriers of BIM application for SMFEs.

**Figure 10:** Level division for enterprise improvement.

**Table 1:** Classified keywords and frequency in the total list of barriers.

Title	Keywords	Frequency
Software	software\cost\pay\data\hardware	39
People	aware(ness)\knowledge\skill(s)\feedback\reluctant(ance)\refuse\stakeholder\employee	43
Organization	training\risk\time\organizational\collaboration\professors\lectures	74
Environment	law\clients\external\standards\assistant(ance)\resource\goverment\guide(line)\ regulation\protect	64

**Table 2:** Associated word according to barrier classification.

Category	Associated words
Software	Cost + high
	Software + training
	Match + hardware
	Interoperability + abroad
	Quality + model

People	Reluctant + change
	Manager + scheduling
	Knowledge + experience
	Support + applicable + attitude
	Participants + negative + attitude
	Integration + collaboration

Organization	Support + training
	Culture + shared
	experts/professor + invest
	Organizational + collaboration
	Change + structure

Environment	Standard + security
	Standard + guidance
	demand/need + client
	Support + government
	Regulation + contract

**Table 3:** Profile of respondents.

Expert	Occupation	Employer	Years of work experience in construction	Years of experience in fire protection engineering
A	Technical support	Construction company	8	5
B	Electrical engineer	Device supplier	20	18
C	Middle manager	Construction company	15	10
D	Vice-general manager	Design company	32	22
E	General manager	Construction company	25	11

**Table 4:** List of the main barriers.

Key factors	Code	Subfactor	Reference	Summary and evaluation
Software	B1	High cost of BIM software	[5, 6, 10, 13–15]	BIM software carries the construction of architectural models in projects, engineering scheduling based on construction information, and the overall communication and coordination functions of the construction team. However, the high cost, high technical requirements, and matching obstacles of BIM professional software are hindering the above functions.
	B2	Lack of domestic-oriented BIM tools	[9, 16–18]	
	B3	High cost of supporting hardware upgrades required	[4, 9, 10, 15–17, 19–23]	
	B4	Lack of suitable simulation models for fire protection engineering	Interview	

People	B5	Top managers are not adapting to the new requirements for coordination and scheduling capabilities	[24–26]	People in construction projects include all stakeholders (e.g., clients, contractor, and architects), employees, and managers of construction companies. Psychological factors and decision-makings have an impact on the technology transformation relevant to BIM in the company.
	B6	Relevant personnel reluctant to change	[17, 18, 23, 25–30]	
	B7	Lack of knowledge and experience in applying BIM	[9, 16, 19, 21, 25, 30]	
	B8	Low level of cross-functional coordination and collaboration	[16, 20, 24–26, 31–33]	

Organization	B9	Lack of funding support for proper BIM training	[16, 17, 19, 21–23, 25, 34]	Organizational factors are considered to be related to the capabilities of enterprises. Cash flow, organizational culture, and cross-organizational collaboration are affecting the ability of organizations to apply BIM. This part focuses on the overall behavior and competitiveness of the enterprise in the market.
	B10	Lack of organizational culture support (a shared vision for the BIM application)	[9, 25, 31, 32]	
	B11	Ambiguity about the benefits of BIM	[7, 16–19, 21–23, 26, 34]	
	B12	Lack of knowledge and experience in cross-organizational collaboration	[7, 9, 19, 22, 31, 33]	
	B13	Difficulty accepting the instability of business development brought by changes in organizational structure	[25, 26, 32, 33]	
	B14	Lack of investment in BIM experts	[16, 17, 23]	

Environment	B15	Lack of BIM laws and regulations applicable to fire protection discipline	Interview	There has not been a sufficient BIM practical experience in the context of fire protection construction. The inadequate standards, legislation, and guidelines especially adapting BIM for fire protection projects make stakeholders and their organizations challenging in the transformation towards digital-driven industrialization in construction.
	B16	Lack of demand for BIM application from clients	[7, 9, 18, 20, 23, 27, 28, 31]	
	B17	Lack of external support such as funding from local government	[7, 16, 17, 20, 24]	
	B18	Lack of appropriate government regulatory measures	[7, 25, 28]	
	B19	Lack of pilot projects for BIM applied in fire protection projects to learn from	[18, 24, 26]	
	B20	Lack of BIM contract standards suitable for fire protection discipline	[9, 16–18, 22, 23, 27]	

**Table 5:** Structural self-interaction matrix developed.

Barrier	B1	B2	B3	B4	B5	B6	B7	B8	B9	B10	B11	B12	B13	B14	B15	B16	B17	B18	B19	B20
B1	—	*W*	*Y*	*X*	*Z*	*Z*	*Z*	*Z*	*W*	*Z*	*Z*	*Z*	*Z*	*W*	*Z*	*Z*	*X*	*Z*	*W*	*Z*
B2		—	*X*	*Y*	*W*	*Z*	*W*	*W*	*W*	*W*	*Z*	*W*	*W*	*Z*	*Z*	*W*	*W*	*X*	*W*	*W*
B3			—	*X*	*Z*	*Z*	*Z*	*Y*	*Z*	*Z*	*W*	*Z*	*Z*	*W*	*Z*	*Z*	*Z*	*Z*	*Z*	*Z*
B4				—	*X*	*Z*	*X*	*W*	*X*	*Z*	*X*	*W*	*X*	*X*	*X*	*Y*	*Z*	*Z*	*W*	*X*
B5					—	*W*	*W*	*W*	*W*	*X*	*W*	*W*	*Y*	*W*	*X*	*W*	*X*	*Z*	*W*	*W*
B6						—	*Y*	*Y*	*X*	*X*	*X*	*X*	*Y*	*Y*	*Z*	*Z*	*X*	*W*	*W*	*Z*
B7							—	*W*	*X*	*Y*	*W*	*W*	*Y*	*X*	*X*	*W*	*X*	*Z*	*W*	*W*
B8								—	*X*	*X*	*W*	*Y*	*W*	*Z*	*Z*	*W*	*W*	*Z*	*X*	*Z*
B9									—	*X*	*X*	*W*	*W*	*Y*	*W*	*X*	*X*	*W*	*Y*	*Z*
B10										—	*X*	*W*	*W*	*Y*	*X*	*X*	*X*	*X*	*W*	*W*
B11											—	*X*	*W*	*W*	*Z*	*Z*	*X*	*Z*	*W*	*Z*
B12												—	*W*	*Z*	*Z*	*W*	*Z*	*Z*	*W*	*W*
B13													—	*Z*	*Z*	*W*	*Z*	*Z*	*X*	*Z*
B14														—	*W*	*X*	*X*	*Z*	*X*	*Z*
B15															—	*Z*	*Z*	*W*	*Z*	*Y*
B16																—	*W*	*W*	*Y*	*Y*
B17																	—	*W*	*Z*	*Z*
B18																		—	*Z*	*W*
B19																			—	*Z*
B20																				—

**Table 6:** Initial reachability matrix.

Barrier	B1	B2	B3	B4	B5	B6	B7	B8	B9	B10	B11	B12	B13	B14	B15	B16	B17	B18	B19	B20
B1	1	0	0	1	0	0	0	0	1	0	1	0	0	0	0	1	0	0	0	0
B2	1	1	1	1	0	0	1	1	0	0	0	0	0	0	0	0	0	0	0	0
B3	0	0	1	0	0	0	1	0	0	0	1	0	0	0	0	0	0	0	0	0
B4	1	0	0	1	0	0	1	0	0	0	1	0	0	0	0	0	0	0	0	0
B5	0	0	0	0	1	1	0	0	0	0	0	0	1	0	0	0	0	0	0	0
B6	0	0	0	0	0	1	0	0	0	0	0	0	0	0	0	0	0	0	0	0
B7	0	0	0	0	1	1	1	0	0	1	1	0	0	1	0	0	0	0	0	0
B8	0	0	0	0	1	1	0	1	0	0	0	0	0	0	0	0	0	0	0	0
B9	0	0	0	0	0	0	1	1	1	0	0	0	0	0	0	0	0	0	1	0
B10	0	0	0	0	1	1	0	1	1	1	0	0	1	1	0	0	0	0	1	0
B11	0	0	0	0	1	1	1	0	1	1	1	0	0	1	0	0	0	0	0	0
B12	0	0	0	0	1	0	0	0	0	0	0	1	1	0	0	0	0	0	0	0
B13	0	0	0	0	0	1	0	1	0	0	0	0	1	0	0	0	0	0	0	0
B14	0	1	0	0	1	0	0	0	0	0	0	0	0	1	0	0	0	0	0	1
B15	0	1	0	0	0	0	0	0	0	0	0	0	0	0	1	0	0	1	0	1
B16	0	1	0	1	0	0	0	0	1	0	0	0	0	1	0	1	0	0	0	0
B17	1	1	1	1	0	0	1	0	1	0	0	0	0	1	1	0	1	0	0	0
B18	0	0	0	0	0	0	0	0	0	0	0	1	0	0	0	0	0	1	0	0
B19	0	0	0	0	0	0	1	1	0	0	1	1	1	0	0	0	0	0	1	0
B20	0	0	1	0	0	0	0	0	0	0	0	0	0	0	0	0	0	1	0	1

**Table 7:** Replacing rules for converting SSIM to reachability matrix.

SSIM (*i*, *j*)	Reachability matrix	
	(*i*, *j*)	(*j*, *i*)
*W*	1	0
*X*	0	1
*Y*	1	1
*Z*	0	0

**Table 8:** Reachability matrix.

Barrier	B1	B2	B3	B4	B5	B6	B7	B8	B9	B10	B11	B12	B13	B14	B15	B16	B17	B18	B19	B20	Driving power
B1	1	1	1	1	1	1	1	1	1	1	1	1	1	1	0	1	0	1	1	1	18
B2	1	1	1	1	1	1	1	1	1	1	1	1	1	1	0	1	0	1	1	1	18
B3	1	1	1	1	1	1	1	1	1	1	1	1	1	1	0	1	0	1	1	1	18
B4	1	1	1	1	1	1	1	1	1	1	1	1	1	1	0	1	0	1	1	1	18
B5	0	0	0	0	1	1	0	1	0	0	0	0	1	0	0	0	0	0	0	0	4
B6	0	0	0	0	0	1	0	0	0	0	0	0	0	0	0	0	0	0	0	0	1
B7	1	1	1	1	1	1	1	1	1	1	1	1	1	1	0	1	0	1	1	1	18
B8	0	0	0	0	1	1	0	1	0	0	0	0	1	0	0	0	0	0	0	0	4
B9	1	1	1	1	1	1	1	1	1	1	1	1	1	1	0	1	0	1	1	1	18
B10	1	1	1	1	1	1	1	1	1	1	1	1	1	1	0	1	0	1	1	1	18
B11	1	1	1	1	1	1	1	1	1	1	1	1	1	1	0	1	0	1	1	1	18
B12	0	0	0	0	1	1	0	1	0	0	0	1	1	0	0	0	0	0	0	0	5
B13	0	0	0	0	1	1	0	1	0	0	0	0	1	0	0	0	0	0	0	0	4
B14	1	1	1	1	1	1	1	1	1	1	1	1	1	1	0	1	0	1	1	1	18
B15	1	1	1	1	1	1	1	1	1	1	1	1	1	1	1	1	0	1	1	1	19
B16	1	1	1	1	1	1	1	1	1	1	1	1	1	1	0	1	0	1	1	1	18
B17	1	1	1	1	1	1	1	1	1	1	1	1	1	1	1	1	1	1	1	1	20
B18	0	0	0	0	1	1	0	1	0	0	0	1	1	0	0	0	0	1	0	0	6
B19	1	1	1	1	1	1	1	1	1	1	1	1	1	1	0	1	0	1	1	1	18
B20	1	1	1	1	1	1	1	1	1	1	1	1	1	1	0	1	0	1	1	1	18
Dependence power	14	14	14	14	19	20	14	19	14	14	14	16	19	14	2	14	1	15	14	14	

**Table 9:** Results of level partitions.

Barrier	Reachability set	Antecedent set	Intersection	Level
B1	1, 2, 3, 4, 5, 6, 7, 8, 9,10,11,12,13,14,16,18,19,20	1, 2, 3, 4, 7, 9, 10,11,14,15,16,17,19,20	1, 2, 3, 4, 7, 9, 10,11,14,16,19,20	IV
B2	1, 2, 3, 4, 5, 6, 7, 8, 9,10,11,12,13,14,16,18,19,20	1, 2, 3, 4, 7, 9, 10,11,14,15,16,17,19,20	1, 2, 3, 4, 7, 9, 10,11,14,16,19,20	IV
B3	1, 2, 3, 4, 5, 6, 7, 8, 9,10,11,12,13,14,16,18,19,20	1, 2, 3, 4, 7, 9, 10,11,14,15,16,17,19,20	1, 2, 3, 4, 7, 9, 10,11,14,16,19,20	IV
B4	1, 2, 3, 4, 5, 6, 7, 8, 9,10,11,12,13,14,16,18,19,20	1, 2, 3, 4, 7, 9, 10,11,14,15,16,17,19,20	1, 2, 3, 4, 7, 9, 10,11,14,16,19,20	IV
B5	5, 6, 8, 13	1, 2, 3, 4, 5, 7, 8, 9, 10,11,12,13,14,15,16,17,18,19,20	8, 5, 13	II
B6	6	1, 2, 3, 4, 5, 6, 7, 8, 9,10,11,12,13,14,15,16,17,18,19,20	6	I
B7	1, 2, 3, 4, 5, 6, 7, 8, 9,10,11,12,13,14,16,18,19,20	1, 2, 3, 4, 7, 9, 10,11,14,15,16,17,19,20	1, 2, 3, 4, 7, 9, 10,11,14,16,19,20	IV
B8	5, 6, 8, 13	1, 2, 3, 4, 5, 7, 8, 9, 10,11,12,13,14,15,16,17,18,19,20	8, 5, 13	II
B9	1, 2, 3, 4, 5, 6, 7, 8, 9,10,11,12,13,14,16,18,19,20	1, 2, 3, 4, 7, 9, 10,11,14,15,16,17,19,20	1, 2, 3, 4, 7, 9, 10,11,14,16,19,20	IV
B10	1, 2, 3, 4, 5, 6, 7, 8, 9,10,11,12,13,14,16,18,19,20	1, 2, 3, 4, 7, 9, 10,11,14,15,16,17,19,20	1, 2, 3, 4, 7, 9, 10,11,14,16,19,20	IV
B11	1, 2, 3, 4, 5, 6, 7, 8, 9,10,11,12,13,14,16,18,19,20	1, 2, 3, 4, 7, 9, 10,11,14,15,16,17,19,20	1, 2, 3, 4, 7, 9, 10,11,14,16,19,20	IV
B12	5, 6, 8,12,13	1, 2, 3, 4, 7, 9, 10,11,12,14,15,16,17,18,19,20	12	III
B13	5, 6, 8, 13	1, 2, 3, 4, 5, 7, 8, 9, 10,11,12,13,14,15,16,17,18,19,20	8, 5, 13	II
B14	1, 2, 3, 4, 5, 6, 7, 8, 9,10,11,12,13,14,16,18,19,20	1, 2, 3, 4, 7, 9, 10,11,14,15,16,17,19,20	1, 2, 3, 4, 7, 9, 10,11,14,16,19,20	IV
B15	1, 2, 3, 4, 5, 6, 7, 8, 9,10,11,12,13,14,15,16,18,19,20	15, 17	15	V
B16	1, 2, 3, 4, 5, 6, 7, 8, 9,10,11,12,13,14,16,18,19,20	1, 2, 3, 4, 7, 9, 10,11,14,15,16,17,19,20	1, 2, 3, 4, 7, 9, 10,11,14,16,19,20	IV
B17	1, 2, 3, 4, 5, 6, 7, 8, 9,10,11,12,13,14,15,16,17,18,19,20	17	17	V
B18	5, 6, 8,12,13,18	1, 2, 3, 4, 7, 9, 10,11,14,15,16,17,18,19,20	18	III
B19	1, 2, 3, 4, 5, 6, 7, 8, 9,10,11,12,13,14,16,18,19,20	1, 2, 3, 4, 7, 9, 10,11,14,15,16,17,19,20	1, 2, 3, 4, 7, 9, 10,11,14,16,19,20	IV
B20	1, 2, 3, 4, 5, 6, 7, 8, 9,10,11,12,13,14,16,18,19,20	1, 2, 3, 4, 7, 9, 10,11,14,15,16,17,19,20	1, 2, 3, 4, 7, 9, 10,11,14,16,19,20	IV

Numbers represent an element, such as 2 represents the second element.

## Data Availability

All data used are included in the manuscript.
